# Computerized Tomography Image Feature under Convolutional Neural Network Algorithm Evaluated for Therapeutic Effect of Clarithromycin Combined with Salmeterol/Fluticasone on Chronic Obstructive Pulmonary Disease

**DOI:** 10.1155/2021/8563181

**Published:** 2021-08-02

**Authors:** Guoping Luo, Anqi Lin, Zhaoqiang Yang, Yujian Chen, Cuiying Mo

**Affiliations:** ^1^Department of Respiration, Shunde Hospital of Guangzhou University of Traditional Chinese Medicine, Shunde District, Foshan City 528300, Guangdong Province, China; ^2^Psychosomatic Medicine, Wuzhongpei Memorial Hospital, Shunde District, Foshan City 528300, Guangdong Province, China

## Abstract

This study was to explore the use of convolutional neural network (CNN) for the classification and recognition of computerized tomography (CT) images of chronic obstructive pulmonary disease (COPD) and the therapeutic effect of clarithromycin combined with salmeterol/fluticasone. First, the clinical data of COPD patients treated in hospital from September 2018 to December 2020 were collected, and CT and X-ray images were also collected. CT-CNN and X ray-CNN single modal models were constructed based on the LeNet-5 model. The randomized fusion algorithm was introduced to construct a fused CNN model for the diagnosis of COPD patients, and the recognition effect of the model was verified. Subsequently, the three-dimensional reconstruction of the patient's bronchus was performed using the classified CT images, and the changes of CT quantitative parameters in COPD patients were compared and analyzed. Finally, COPD patients were treated with salmeterol/fluticasone (COPD-C) and combined with clarithromycin (COPD-T). In addition, the differences between patients' lung function indexes, blood gas indexes, St. George respiratory questionnaire (SGRQ) scores, and the number of acute exacerbations (AECOPD) before and after treatment were evaluated. The results showed that the randomized fusion model under different iteration times and batch sizes always had the highest recognition rate, sensitivity, and specificity compared to the two single modal CNN models, but it also had longer training time. After CT images were used to quantitatively evaluate the changes of the patient's bronchus, it was found that the area of the upper and lower lung lobes of the affected side of COPD patients and the ratio of the area of the tube wall to the bronchus were significantly changed. The lung function, blood gas index, and SGRQ score of COPD-T patients were significantly improved compared with the COPD-C group (*P* < 0.05), but there was no considerable difference in AECOPD (*P* > 0.05). In summary, the randomized fusion-based CNN model can improve the recognition rate of COPD, and salmeterol/fluticasone combined with clarithromycin therapy can significantly improve the clinical treatment effect of COPD patients.

## 1. Introduction

Chronic obstructive pulmonary disease (COPD) is a disease with a high prevalence and fatality rate in the world. The quality of life of patients with advanced COPD will be significantly reduced, and long-term oxygen therapy and drug treatment are required, which brings a huge burden to the patient's family [1]. The main pathological changes of COPD are lung parenchymal damage and airway damage, among which the main manifestation of lung parenchymal damage is emphysema, and airway damage is classified into central trachea or small trachea injury [2]. The main clinical methods used to detect COPD small airway damage are computerized tomography (CT) and pulmonary function test (PFT) examinations. PFT examination focuses on spirometry, single breathing method, repeated breathing method, and pulse oscillation method, which is the gold standard for clinical diagnosis and grading of COPD [3, 4].

With the improvement of the computing level, deep learning has harvested excellent results in many fields such as speech recognition, and medical image classification based on deep learning has gradually replaced manual operation [5, 6]. The deep learning method mostly used in the field of medical imaging is convolutional neural network (CNN). The model contains special structures such as convolutional layer and pooling layer, which significantly improve the classification and recognition accuracy of the model [7].

At present, anti-inflammatory therapy is of great significance in the treatment of COPD disease. The drugs used in anti-inflammatory treatment are mainly glucocorticoids. Most studies recommend the use of salmeterol/fluticasone inhalation [8]. However, the drug used in the treatment of COPD can increase the risk of pneumonia, and it is difficult for most patients to accept it. In recent years, studies found that macrolide antibiotics have certain antibacterial effects, as well as anti-inflammatory and immunomodulatory effects, which have good results in the treatment of chronic inflammatory reactive lung diseases [9]. Studies have shown that oral clarithromycin combined with inhaled salmeterol in the treatment of chronic pulmonary obstruction has a good effect and high safety.

A model for image classification and recognition of COPD patients was proposed based on the CNN model, and the morphological changes of the small trachea of COPD patients were quantitatively analyzed based on the CT images after classification. Moreover, the therapeutic effects of inhaled corticosteroids on COPD patients were compared and analyzed, aiming to provide a reference for improving the clinical diagnosis rate of COPD and improving the treatment effect of patients.

## 2. Materials and Methods

### 2.1. Research Subjects

The clinical data of 58 patients with COPD who were treated in hospital from September 2018 to December 2020 were collected. COPD patients met the diagnostic criteria of the *Guidelines for the Diagnosis of Chronic Obstructive Pulmonary Disease Pulmonary Diseases* (2013 revision). Among them, 35 were males and 23 were females, aged 44 to 63 years old. The 50 healthy people who had undergone physical examinations in the hospital served as controls. Among them, 32 were males and 18 were females, aged 42–61 years old. Exclusion criteria: (i) those with bronchiectasis, pulmonary bullae, pulmonary fibrosis, and pulmonary space-occupying diseases that affect lung function; (ii) those with organic heart disease; (iii) those underwent chest surgery in history; and (iv) those who suffered from other diseases that restrict respiratory movement. The experimental procedure of this study had been approved by the Medical Ethics Committee of the Hospital, and all subjects had signed written informed consent.

### 2.2. Lung Function and Blood Gas Index Measurement

All subjects were required to complete pulmonary function measurements within seven days before and after the CT scan. Measurement function parameters included forced expiration in the first second (FEV1), forced expiratory volume percentage (FEV%), and forced expiratory volume in the first second/forced vital capacity (FEV1/FVC%). In addition, the PaO_2_ and PaCO_2_ blood gas indexes in the arterial blood of the patient were measured. All patients needed to undergo pulmonary function tests and be able to meet the criteria for diagnosing COPD.

### 2.3. CT Scan Process

The patient's chest image was scanned using 64-slice MSCT, and the patient underwent breathing training before the scan. During the examination, the patient was placed in the supine position for CT scan, and the whole lung was examined when the patient took a deep breath and reached the optimal inflatable state after holding his breath. Scanning parameters were set as follows: 0.875 pitch, 38 × 38 cm field of view, 512 × 512 matrix, 1500 window width, −650U window level, 0.5 cm layer thickness, and 0.5 cm layer spacing. CT image reconstruction was performed using the standard CT reconstruction algorithm, and the layer thickness was set as 0.625 mm and the layer spacing was set as 0.625 mm. The reconstructed CT images were uploaded to the workstation, and Thoracic VCAR Airway Analysis software was used to measure the airway. The lumen diameter, area ratio of trachea to bronchial wall, wall thickness, and diameter ratio of the air duct (trachea, main bronchus, apical segment of upper lobe/posterior segment/anterior segment, etc.) were measured.

### 2.4. COPD Image Classification and Recognition Based on CNN

Firstly, a single mode CNN model was constructed to extract the feature vectors of the CNN full connection layer, and a randomized function was constructed. The data of the full connection layer of different modes were randomly fused, and the fused feature recognition was used for the classification of COPD images, so as to improve the image classification effect.

#### 2.4.1. Multimodal Feature Fusion Based on Stochastic Fusion

The methods of multimodal feature fusion recognition designed in this study were (i) the processing of CT images and chest X-ray images; (ii) multimodal lung image features extracted using LeNet-5 network; (iii) stochastic function used for the fusion of parallel multimodal features and the reconstruction of target features in the same dimension; and (iv) the full connection layer and the classification layer added to carry out the regression training of the network, so as to get the results after classification.

The basic structure of the LeNet-5 network model [10] is shown in Figure 1, and the algorithm flow of using randomized fusion algorithm combined with multimodal CNN lung image recognition is shown in Figure 2.

The LeNet-5 model was employed to extract the features of the image, and then the model's own parameter transfer learning ability was adopted to adjust the parameters of the model. The size of the training data needed to be randomly selected when the model was trained, and the data were sequentially input into the model for training according to the set batches. At the same time, the weight value and bias of the model needed to be adjusted. It is required to input all the data in the test set into the network when the model was tested. The network parameters were set to the optimal number of adoption during training, and the classifier was used to recognize COPD. The network structure constructed in this study is shown in Figure 3.

From Figure 3, there were two CNN network models designed, namely, CT-CNN and X ray-CNN, and the specific parameter settings of the network are shown in Table 1. There were certain differences in the parameters between different network layers. The input data of the input layer needed to be randomly selected from the training set according to the size of the batch and form a vector with a certain dimension. The convolutional layer needed to initialize the convolution kernel size, weight value, and bias. Then, the convolution kernel and the input data were convolved to enhance the feature matrix in the image and remove noise. The activation function used was the Sigmoid function [11], and the pooling operation was an average pooling operation. Rand random function [12] was used to randomize the feature vector, weight, and bias in the last layer of the fully connected layer.

### 2.5. Treatment Methods

58 COPD patients were randomly divided into two groups—the control group (COPD-C) and the treatment group (COPD-T)—with 28 and 30 patients, respectively. Patients in the COPD-C group inhaled 50/250 *μ*g of salmeterol/fluticasone twice a day. Patients in the COPD-T group were given oral clarithromycin sustained-release tablets for combination therapy based on the inhalation of salmeterol/fluticasone. In addition, 0.5 g clarithromycin sustained-release tablets should be taken orally once a day, and 50/250 *μ*g salmeterol/fluticasone should be inhaled twice a day. All patients took 10 days as a course of treatment and cannot take *β*-agonist and hormone inhalation therapy within 15 days before receiving the treatment. After treatment, a 3-month follow-up was conducted to record the patient's drug use, changes in the condition, the number of acute exacerbations, and adverse reactions.

### 2.6. Evaluation Indexes

The number of acute exacerbations of COPD (AECOPD) in the patient was recorded. St. George Respiratory Questionnaire (SGRQ) score sheet was used to evaluate the patient. The lower the score is, the better the patient's function is, and it was meaningful to reduce the total score of SGRQ by more than 4 points in clinical practice. After treatment, the lung function indexes were evaluated, as shown in Section 2.2. Moreover, the probability of adverse reactions in patients after treatment was recorded.

The recognition rate, sensitivity, and specificity were calculated to evaluate the construction model. The calculation equations for different indexes were as follows:

(1) $$\begin{array}{c} \mathrm{recognition}=\frac{\mathrm{TP+TN}}{\mathrm{TP+TN+FP+FN}},\\ \mathrm{sensitivity}=\frac{\mathrm{TP}}{\mathrm{TP+FN}},\\ \mathrm{specificity}=\frac{\mathrm{TN}}{\mathrm{TN+FP}}. \end{array}$$

TP is true positive, FP is false positive, TN is true negative, and FN is false negative.

### 2.7. Statistical Methods

Subsequently, SPSS 19.0 was used for statistical analysis. Measurement data were expressed as mean ± standard deviation, and independent sample *t*-test was used for difference comparison. Count data were expressed by frequency (percentage), and the difference was compared using chi-square test or Fisher's test. *P* < 0.05 means that the difference was statistically significant.

## 3. Results

### 3.1. Model Training for CT Image Classification

The parameter transfer method was adopted to train the constructed CNN model. Comparison and analysis of the differences among model recognition rate, training time, sensitivity, and specificity under different iteration times are shown in Figure 4. From Figure 4(a), as the number of iterations increased, the recognition rates of CT-CNN, X ray-CNN, and randomized fusion showed a gradual increase trend. However, the recognition rate of the randomized fusion model was always higher than that of other models. The recognition rates of CT-CNN, X ray-CNN, and randomized fusion under the maximum number of iterations were 95.8%, 99.0%, and 99.8%, respectively. From Figure 4(b), as the number of iterations increased, the training times of different models showed a gradual increase trend. Among them, the training time of the randomized fusion model was always the longest, and there was no significant difference between the training time of the CT-CNN and X ray-CNN models. From Figure 4(c), the recognition sensitivity of different models showed different changes as the number of iterations increased. The sensitivities of CT-CNN, X ray-CNN, and randomized fusion at the maximum number of iterations were 83.4%, 95.8%, and 99.5%, respectively. From Figure 4(d), as the number of iterations increased, the recognition specificity of different models gradually increased. CT-CNN, X ray-CNN, and the recognition specificity of the randomized fusion model was 99.6%, 95.8%, and 100.0%, respectively.

The differences of model recognition rate, training time, sensitivity, and specificity under different batch sizes are shown in Figure 5. From Figures 5(a) and 5(b), as the training batch increased, the recognition rate and training time of CT-CNN, X ray-CNN, and randomized fusion models showed a gradual decline. When the maximum training batch was reached, the recognition rates were 97.4%, 96.0%, and 98.6%, and the training time was 67.2 s, 63.4%, and 193.6 s, respectively. Among them, the randomized fusion model had the highest recognition rate and the longest training time. From Figure 5(c), with the increase of training batches, the recognition sensitivity of different models first increased and then decreased. When the training batch reached 100, the sensitivity was the lowest, but the randomized fusion model had the highest sensitivity compared with the CT-CNN and X ray-CNN models. From Figure 5(d), the recognition specificity of each model changed with the training batch, and the recognition specificity of the randomized fusion model was always the highest.

### 3.2. Quantitative Analysis of CT Bronchus in Patients with COPD

The differences between the baseline data of the healthy control group and COPD patients are shown in Table 2. There was no significant difference in average age, sex ratio, and BMI indexes between the control group and COPD group (*P* > 0.05

The difference between the LA and WA% of the bronchi of the upper and lower lobe of the affected lung in the control group and the COPD group was evaluated (Figure 6). CT images classified by CNN were used to reconstruct the patient's bronchi in three dimensions. From Figure 6(a), the lung bronchus of the COPD group showed obvious obstruction. From Figures 6(b) and 6(c), the upper lobe of the affected side of the COPD group had significantly increased LA in the upper lobe of the lung and significantly reduced LA in the 5 and 6 levels compared with the control group (*P* < 0.05), and WA% in the 5 and 6 levels greatly increased (*P* < 0.05). From Figures 6(d) and 6(e), the LA of the lower lobe of the affected lung in the COPD group was significantly reduced in grade 6, 7, and 8, while the WA% was significantly increased compared with the control group (*P* < 0.05).

### 3.3. Analysis of the Treatment Effect of Patients with COPD

#### 3.3.1. Changes in Lung Function and Blood Gas Indexes in Patients with COPD

The changes in lung function and blood gas indexes of patients before and after treatment are compared in Figure 7. There was no significant difference in the FEV1, FVC, FEV1/FVC, PaO_2_, and PaCO_2_ between patients in COPD-C group and COPD-T group before treatment (*P* > 0.05). After treatment, compared with patients in the COPD-C group, FEV1, FVC, FEV1/FVC, and PaO_2_ in COPD-T patients increased significantly, and PaCO_2_ decreased significantly (*P* < 0.05).

#### 3.3.2. Comparison of Differences in Other Indexes of COPD Patients after Treatment

The difference of the SGRQ scores before and after treatment and the number of AECOPD during treatment between the two groups of patients is compared in Figure 8. From Figure 8(a), there was no considerable difference in SGRQ scores between the two groups before treatment (*P* > 0.05). Compared with the COPD-C group, the SGRQ score of the COPD-T group was significantly reduced after treatment (*P* < 0.05). From Figure 8(b), there was no great difference in the number of AECOPDs between the two groups of patients during treatment (*P* > 0.05).

## 4. Discussion

The CNN model is a feed forward neural network, and it is a multilayer perceptron model constructed to recognize two-dimensional and above images [13,14]. The current CNN model includes LeNet and AlexNet models, among which the LeNet-5 model is relatively mature, and the network structure is simpler [15,16]. To improve the clinical diagnosis rate of COPD, two single-modal CNN models were constructed using patient CT images and X-ray images. Then, the randomized fusion algorithm was adopted to fuse the CT-CNN and X ray-CNN models to obtain a randomized fusion model. The model recognition effect was evaluated, and the test results showed that the recognition rate, sensitivity, and specificity of the randomized fusion model increased greatly. It showed that the use of single-modal CNN model fusion for feature extraction of patient images can improve the effect of patient feature extraction and classification and recognition.

COPD is a common and frequent disease in respiratory system diseases. Clarithromycin combined with salmeterol and fluticasone has a significant effect in the treatment of chronic pulmonary obstruction. Patients with stable chronic obstructive pulmonary disease have a relatively stable condition. However, if patients with acute-onset chronic obstructive pulmonary disease cannot be further treated, their condition will become worse and cause respiratory failure, hypoxemia, and other serious complications [17,18]. The results of Renkema et al. [19] showed that the airway hyper-responsiveness of nonallergic patients with chronic obstructive malignant disease increased over time. In this research, the patient's affected lung lobe bronchus was scanned for quantitative evaluation. The results showed that COPD patients had significant changes in LA and WA% of grades 5∼6 bronchus in the upper lobes of the lung and had LA and WA% of grades 6∼8 in the lower lobes of the lung compared with healthy people. Studies revealed that, with the aggravation of COPD disease, LA gradually decreases, while WA% gradually increases.

Due to the relatively poor diffusion function of small airways, the inflammatory response of COPD is determined by the activation of respiratory epithelial cells and macrophages. Therefore, the bronchial tube wall is thickened, and the lumen is narrowed in patients with COPD. Combined with the results obtained in this study, it was suggested that LA and WA% can be used to quantitatively assess the morphological changes of the bronchus in patients with COPD and can also be used for the diagnosis of COPD.

Salmeterol is a long-acting *β*2 receptor agonist, which is used for the relaxation of airway smooth muscle and can also inhibit the release of inflammatory mediators [20]. Fluticasone is an inhaled glucocorticoid, which acts on glucocorticoid receptors and increases the sensitivity of *β*2 receptors, thereby delaying airway remodeling. The results of Jin [21] and other studies showed that patients with chronic obstructive disease had higher serum levels, and the impairment of lung function was related to symptoms such as serum levels and dyspnea. In addition to antibacterial properties, clarithromycin also has anti-inflammatory and immunomodulatory effects. Salmeterol/fluticasone and clarithromycin were combined for the treatment of COPD in this research. The results showed that salmeterol/fluticasone and combined clarithromycin treatment can significantly reduce the SGRQ score of COPD patients. It was proved that salmeterol/fluticasone combined with clarithromycin treatment can significantly improve the lung function of COPD patients.

## 5. Conclusion

The randomization and fusion of the single-modal CNN model can improve the recognition effect of COPD, and CT quantitative indexes can be used for the diagnosis of COPD. Moreover, combined treatment of salmeterol/fluticasone and clarithromycin can significantly improve the lung function of COPD patients and enhance the clinical treatment effect. However, this study only analyzed the CT image and X-ray image of COPD patients based on the constructed CNN model. Follow-up work should combine it with clinical biology and other indexes to comprehensively compare the differences between the diagnosis rates of COPD. In short, this study can provide a reference for improving the clinical diagnosis and treatment of COPD.

## Figures and Tables

**Figure 1:** The basic structure of the LeNet-5 model. FC is the fully connected layer; Softmax is the activation function.

**Figure 2:** Multimodal CNN lung image recognition process based on randomized fusion algorithm.

**Figure 3:** The basic structure of the CNN model.

**Figure 4:** Changes in the recognition efficiency of single-modal CNN and randomized fusion models under different iteration times. (a) The recognition rate. (b) The training time. (c) The recognition sensitivity. (d) The recognition specificity.

**Figure 5:** Changes in the recognition efficiency of single-modal CNN and randomized fusion models under different batches. (a) The recognition rate. (b) The training time. (c) The recognition sensitivity. (d) The recognition specificity.

**Figure 6:** Comparison of quantitative parameters of bronchus between normal and COPD patients based on CT reconstruction. (a) The three-dimensional reconstruction of the bronchial CT image. (b) The LA detection of the upper lobe of the affected side of the lung. (c) The WA% detection of the upper lobe of the affected side of the lung. (d) The LA detection of the lower lobe of the affected side of the lung. (e) The WA% detection of the lower lobe of the affected side of the lung. ^*∗*^*P* < 0.05.

**Figure 7:** Comparison of lung function and blood gas indexes between two groups of COPD patients before and after treatment. (a) FEV1. (b) FVC. (c) FEV1/FVC. (d) PaO_2_. (e) PaCO_2_. ^*∗*^*P* < 0.05.

**Figure 8:** Comparison of SGRQ scores and AECOPD times between two groups of COPD patients before and after treatment. (a) The comparison of SGRQ scores before and after treatment. (b) The comparison of AECOPD times during treatment. ^*∗*^*P* < 0.05.

**Table 1:** Structure and parameter setting of the CNN model.

Framework	Input	Convolution		Pooling		Structure				
		Convolution kernel	Step size	Size	Step size	Convolutional layer	Sigmoid	Average pooling	Fc	Rand
Input layer	28 × 28	—	—	—	—	—	—	—	—	—
Conv (1)	24 × 24 × 6	3 × 3	1	2 × 2	2	+	+	+	—	—
Conv (2)	8 × 8 × 12	3 × 3	1	2 × 2	2	+	+	+	—	—
Fc (1)	4 × 4 × 12	1 × 1	—	—	—	—	+	—	+	—
Fc (2)	192 × 3	1 × 1	—	—	—	—	+	—	+	+

*Note.* + means yes; —means no.

**Table 2:** Comparison of baseline data of patients.

Item	Control group (*n* = 50)	COPD group (*n* = 58)	Statistics	*P*
Age (years old)	56.7 ± 5.7	58.3 ± 6.2	*t* = 0.133	0.883
Male (cases/%)	32/64.0	35/60.3	*χ*^2^ = 1.204	0.559
BMI (kg/m^2^)	21.4 ± 1.6	21.6 ± 1.4	*t* = -2.125	0.936

BMI: body mass index.

## Data Availability

The data used to support the findings of this study are included within the article.
